The article "The candidate tumor suppressor gene ECRG4 inhibits cancer cells migration and invasion in esophageal carcinoma" was retracted in 2011. Reasons: duplicated text; duplicate publication.

# The candidate tumor suppressor gene ECRG4 inhibits cancer cells migration and invasion in esophageal carcinoma

**DOI:** 10.1186/1756-9966-29-133

**Published:** 2010-10-11

**Authors:** Linwei Li, Chunpeng Zhang, Xiaoyan Li, ShihHsin Lu, Yun Zhou

**Affiliations:** 1 Oncology Department, Henan Provincial People's Hospital, Zhengzhou 450003, PR China; 2 State Key Laboratory of Molecular Oncology and Department of Etiology and Carcinogenesis, Cancer Institute & Hospital, Chinese Academy of Medical Sciences & Peking Union Medical College, Beijing 100021, PR China

## Abstract

**Background:**

The esophageal cancer related gene 4 (ECRG4) was initially identified and cloned in our laboratory from human normal esophageal epithelium (GenBank accession no.AF325503). ECRG4 was a new tumor suppressor gene in esophageal squamous cell carcinoma (ESCC) associated with prognosis. In this study, we investigated the novel tumor-suppressing function of ECRG4 in cancer cell migration, invasion, adhesion and cell cycle regulation in ESCC.

**Methods:**

Transwell and Boyden chamber experiments were utilized to examined the effects of ECRG4 expression on ESCC cells migration, invasion and adhesion. And flow cytometric analysis was used to observe the impact of ECRG4 expression on cell cycle regulation. Finally, the expression levels of cell cycle regulating proteins p53 and p21 in human ESCC cells transfected with ECRG4 gene were evaluated by Western blotting.

**Results:**

The restoration of ECRG4 expression in ESCC cells inhibited cancer cells migration and invasion (*P *< 0.05), which did not affect cell adhesion capacity (*P *> 0.05). Furthermore, ECRG4 could cause cell cycle G1 phase arrest in ESCC (*P *< 0.05), through inducing the increased expression of p53 and p21 proteins.

**Conclusion:**

ECRG4 is a candidate tumor suppressor gene which suppressed tumor cells migration and invasion without affecting cell adhesion ability in ESCC. Furthermore, ECRG4 might cause cell cycle G1 phase block possibly through inducing the increased expression of p53 and p21 proteins in ESCC.

## Introduction

Esophageal carcinoma ranks 7^th ^and 6^th ^in terms of cancer incidence and mortality rate worldwide, respectively [1]. Moreover, nearly 50% of esophageal carcinoma cases in the world occurred in China [2]. Esophageal squamous cell carcinoma (ESCC), which is the most common histological subtype, accounts for ~90% of all esophageal cancers diagnosed in China each year. Despite advances in clinical comprehensive treatment, ESCC prognosis remains poor due to its diffuse and invasive nature. To date, the molecular pathogenesis of ESCC is still unclear [3,4].

The ECRG4 gene (GenBank accession no. AF325503) was initially identified and cloned in our laboratory from human normal esophageal epithelium [5,6]. Our previous results demonstrated that ECRG4 protein was an independent prognostic factor for ESCC, and the low expression of ECRG4 protein in patients with ESCC was associated with poor prognosis [7,8]. Furthermore, overexpression of ECRG4 gene in ESCC cells inhibited tumor cells growth *in vitro *and *in vivo *[7,8].

The article "The candidate tumor suppressor gene ECRG4 inhibits cancer cells migration and invasion in esophageal carcinoma" was retracted in 2011. Reasons: duplicated text; duplicate publication.

In the present study, we further examined the tumor-suppressing function of ECRG4 gene, in terms of cell migration and invasion, and explored possible molecular mechanism in ESCC.

## Materials and methods

### Construction of eukaryotic expression vector and stable transfection

The coding region of ECRG4 cDNA was subcloned into constitutive mammalian expression vector pcDNA3.1 (Invitrogen). The cDNA was then fully sequenced to ensure that no mutation was introduced during the PCR amplification. The resulting plasmid construct was named pcDNA3.1-ECRG4. The human esophageal squamous cell line EC9706 was established and studied by Han *et al *[9]. EC9706 cells were seeded in 6-cm dishes at 5×10^5 ^cells/dish and transfected with pcDNA3.1-ECRG4 and pcDNA3.1 using lipofectamine™2000 (Invitrogen), according to the manufacturer's protocol. After culturing in medium containing 400 μg/ml of geneticin (Invitrogen) for 3 weeks, individual clones were isolated. Clones that expressed the ECRG4 cDNA coding region were maintained in medium containing 200 μg/ml of geneticin and used for further experiments.

### Cell proliferation assay

EC9706 cells (pcDNA3.1 and pcDNA3.1-ECRGR4) were seeded into 96-well plates (1.5 × 10^3 ^cells/well). After culturing for various durations, cell proliferation was evaluated by thiazolyl blue tetrazolium bromide (MTT) assay, according to the manufacturer's protocol (Sigma-Aldrich Co., St. Louis, MO, USA). In brief, 10 μl MTT solution (5 mg/ml) was added to each well, then the cells were cultured for another 4 hours at 37°C, and 100 μl DMSO was added to each well and mix vigorously to solubilize colored crystals produced within the living cells. The absorbance at 570 nm was measured by using a multi-well scanning spectrophotometer Victor 3.

### *In vitro *cell migration and invasion assay

Cells growing in the log phase were treated with trypsin and re-suspended as single-cell solutions. A total of 1 × 10^5 ^cells in 0.5 ml of serum-free RPMI 1640 medium were seeded on a 8 μm-pore polycarbonate membrane Boyden chambers insert in a transwell apparatus(Costar, Cambridge, MA), either coated with or without Matrigel(BD Biosciences, San Jose, CA). 600 μl RPMI1640 containing 20% FBS was added to the lower chamber. After the cells were incubated for 12-24 hours at 37°C in a 5% CO_2 _incubator, cells on the top surface of the insert were removed by wiping with a cotton swab. Cells that migrated to the bottom surface of the insert were fixed in 100% methanol for 2 minutes, stained in 0.5% crystal violet for 2 min, rinsed in PBS and then subjected to microscopic inspection (×200). Values for invasion and migration were obtained by counting five fields per membrane and represent the average of three independent experiments.

The article "The candidate tumor suppressor gene ECRG4 inhibits cancer cells migration and invasion in esophageal carcinoma" was retracted in 2011. Reasons: duplicated text; duplicate publication.

### Cell adhesion assay

Cells were plated on 100 ng/μl Matrigel-coated 96-well plates at a density of 5 × 10^4 ^per well. The cells were incubated at 37°C for 30, 60, and 90 minutes in a 5% CO_2 _incubator, respectively. Nonattached cells were removed by PBS washings for three times. Attached cells were analyzed by 3-(4,5-dimethylthiazol-2-yl)-5-(3-carboxymethoxyphenyl)-2-(4-sulfophenyl)-2H-tetrazolium (MTS; Promega, Madison, WI) assay according to the user manual. The mean absorbance values for statistical analysis represent the average of three independent experiments.

### Western blot analysis

Whole-cell lysates of EC9706 cells were prepared by incubating cells in RIPA buffer (1% NP-40; 0.5% sodium deoxycholate; 0.1% SDS; 50 mM Tris-HCl [pH 7.5]) containing protease inhibitors. Cell lysates were centrifuged at 10,000 g for 10 minutes at 4°C. The supernatant was collected, and the protein concentration was measured using the BCA ™ Protein Assay Kit (Pierce). Proteins (40 ug) in cell lysates or culture media were separated by 10-15% SDS-polyacrylamide gel electrophoresis and transferred onto PVDF membrane. The membranes were blocked in TBST (0.2 M NaCl; 10 mM Tris pH7.4; 0.2% Tween20)/5% skim milk for 2 hours at room temperature and then incubated with primary antibodies in TBST/5% skim milk. The primary antibodies used for Western blot analysis were polyclonal rabbit anti-ECRG4 (1:2000) [8], polyclonal rabbit anti-p21(1:4000; Santa Cruz, CA), polyclonal rabbit anti-p53 (1:4000; Santa Cruz, CA), and monoclonal mouse anti-β-actin (1:4000; Santa Cruz, CA). The membranes were then washed three times with TBST, followed by incubation with horseradish peroxidase-conjugated secondary antibody (1:4000) in TBST/5% skim milk. Bound antibody was visualized using ECL detection reagent.

### RT-PCR analysis

Cells were washed with PBS and collected for RT-PCR. The primers designed for ECRG4 were 5'-GGT TCT CCC TCG CAG CAC CT-3' as forward and 5'-CAG CGT GTG GCA AGT CAT GGT TAG-3' as reverse. Thermal cycles were: at 95°C for 2 min, then 30 cycles at 95°C for 30 sec, at 62°C for 30 sec, at 72°C for 1 min followed by extension at 72°C for 7 min [7].

The article "The candidate tumor suppressor gene ECRG4 inhibits cancer cells migration and invasion in esophageal carcinoma" was retracted in 2011. Reasons: duplicated text; duplicate publication.

### Flow cytometric analysis of cell cycle

The transfected cells (pcDNA3.1-ECRG4 and pcDNA3.1) were seeded at a density of 10^6 ^cells/100-mm dish in RPMI-1640 medium with 10% FBS for 48 hours. Then cells were washed with ice-cold PBS, harvested and fixed in 70% ethanol for 30 minutes. Cells were treated with RNase A and stained with 25 μg/ml propidium iodide (PI). Samples were analyzed using a FACScan flow cytometer (Becton Dickinson), according to the manufacturer's protocol. Experiments were performed three times in triplicate. The mean values for statistical analysis represent the average of three independent experiments.

### Statistical analysis

All statistical analysis was performed with the SPSS statistical program (version 13.0). Statistical significance was determined using Student's *t*-tests and analysis of variance. *P *< 0.05 was considered statistically significant.

## Results

### ECRG4 overexpression suppressed cell migration and invasion

The stable-transfected EC9706/pcDNA3.1-ECRG4 cells exhibited detectable ECRG4 mRNA (Figure 1A) and ECRG4 protein expression (Figure 1B), compared with EC9706/pcDNA3.1 cells and EC9706 cells. And the cell growth curve of EC9706/pcDNA3.1-ECRG4 and EC9706/pcDNA3.1 was plotted for further migration-invasion analysis (Figure 1C). To measure the effect of ECRG4 overexpression on tumor cell migration, cells growing in the log phase were collected and cultured on Transwell apparatus. After 12 h incubation, cell migration was significantly decreased in EC9706/pcDNA3.1-ECRG4 group than in control group (*P *< 0.05) (Figure 2). Using Boyden chamber precoated with Matrigel, we examined the effect of ECRG4 overexpression on tumor cell invasion. After 24 h incubation, EC9706/pcDNA3.1-ECRG4 cells showed significantly decreased invasiveness, compared with the EC9706/pcDNA3.1 cells (*P *< 0.05) (Figure 3). These results demonstrated that ECRG4 overexpression reduced the migration and invasion of ESCC cells.

**Figure 1:** **Evaluation of ECRG4 gene expression and cell growth curve of EC9706/pcDNA3.1 and EC9706/pcDNA3.1-ECRG4**. (**A**) ECRG4 mRNA was detected in EC9706/pcDNA3.1-ECRG4 cells by RT-PCR. M: Marker; Lane 1: EC9706/pcDNA3.1; Lane 2: EC9706/pcDNA3.1-ECRG4; Lane 3: EC9706 cells. (**B**) ECRG4 protein (17 KD) was detected in EC9706/pcDNA3.1-ECRG4 cells by Western blot. Lane 1: EC9706 cells; Lane 2: EC9706/pcDNA3.1; Lane 3: EC9706/pcDNA3.1-ECRG4. (**C**) Cell growth curve of EC9706/pcDNA3.1 and EC9706/pcDNA3.1-ECRG4 by MTT assay (*P *< 0.05).

**Figure 2:** **Effect of ECRG4 overexpression on tumor cells migration**. Representative photos and statistic plots of migration assay in EC9706/pcDNA3.1-ECRG4 and EC9706/pcDNA3.1 cells (×200). The number of EC9706/pcDNA3.1-ECRG4 cells transversed the Transwell membrane was decreased compared with that of EC9706/pcDNA3.1 cells (*P *< 0.05). Error bars represent standard deviation from mean value.

The article "The candidate tumor suppressor gene ECRG4 inhibits cancer cells migration and invasion in esophageal carcinoma" was retracted in 2011. Reasons: duplicated text; duplicate publication.

**Figure 3:** **Effect of ECRG4 overexpression on tumor cells invasion**. Representative photos and statistic plots of invasion assay in EC9706/pcDNA3.1-ECRG4 and EC9706/pcDNA3.1 cells (×200). The number of EC9706/pcDNA3.1-ECRG4 cells transversed the Transwell membrane was decreased compared with that of EC9706/pcDNA3.1 cells (*P *< 0.05). Error bars represent standard deviation from mean value.

### The impact of ECRG4 overexpression on cell adhesion capacity

As the apparent ECRG4-induced decrease in migration and invasion could be the result of reduction in adhesion of tumor cells to the substrate, we evaluated cell adhesive ability by measuring the number of cells attached to Matrigel. No significant difference was detected between the two groups by MTS adhesion assay (*P *> 0.05) (Table 1). Therefore, ECRG4 overexpression in EC9706 cells drastically suppressed cancer cells mobility without affecting cell adhesion capacity.

**Table 1:** ECRG4 exerted no significant effect on tumor cells adhesion capacity

Group	30 min	60 min	90 min
EC9706/pcDNA3.1-ECRG4 *	1.268 ± 0.293	1.988 ± 0.341	2.564 ± 0.537
EC9706/pcDNA3.1	1.274 ± 0.247	2.040 ± 0.360	2.531 ± 0.524

* *P *> 0.05, compared with EC9706/pcDNA3.1

### ECRG4 overexpression blocked cell cycle progression

The stable-transfected EC9706/pcDNA3.1-ECRG4 cells exhibited detectable ECRG4 protein expression compared with EC9706/pcDNA3.1 cells, as shown in Figure 1B. The percentages of cells in the G1, S and G_2_/M phase of cell cycle demonstrated that overexpression of ECRG4 in EC9706 cells resulted in an accumulation of cells in G1 phase and a decrease in S and G_2_/M phase compared with EC9706/pcDNA3.1 control cells (*P *< 0.05) (Table 2). Flow cytometric analysis suggested that ECRG4 overexpression could arrest EC9706 cells at the G1/S checkpoint and delay cell cycle into S phase. Consequently, ECRG4 overexpression slowed down cell cycle progression and caused cell cycle G1 phase block.

**Table 2:** ECRG4 overexpression caused cell cycle G1 phase block

Group	G1	S	G2/M
EC9706/pcDNA3.1-ECRG4*	73.7 ± 1.86	14.8 ± 1.13	11.5 ± 0.92
EC9706/pcDNA3.1	59.8 ± 2.06	25.0 ± 1.39	15.2 ± 1.64

* *P *< 0.05, compared with EC9706/pcDNA3.1

### ECRG4 may be involved in p53 pathway

In exploring the molecular mechanism of cell cycle G1 phase block caused by ECRG4 overexpression in EC9706 cells, we found that p53 and p21 protein expression levels were increased in EC9706/pcDNA3.1-ECRG4 cells compared with in EC9706/pcDNA3.1 cells (Figure 4). It indicated that ECRG4 may be involved in p53 pathway in ESCC. ECRG4 might induce p21 upregulation through p53 pathway to block cell cycle progression in ESCC.

The article "The candidate tumor suppressor gene ECRG4 inhibits cancer cells migration and invasion in esophageal carcinoma" was retracted in 2011. Reasons: duplicated text; duplicate publication.

**Figure 4:** **ECRG4 may be involved in p53 pathway**. Representative photos and statistic plots of relative protein expression levels in EC9706/pcDNA3.1-ECRG4 and EC9706/pcDNA3.1. Analysis of cell's total proteins by Western blot showed that p53 and p53 target gene p21 expressions were increased in EC9706/pcDNA3.1-ECRG4 cells compared with in EC9706/pcDNA3.1 cells (*P *< 0.05). Lane 1: EC9706/pcDNA3.1-ECRG4; Lane 2: EC9706/pcDNA3.1. *, *P *< 0.05, compared with EC9706/pcDNA3.1.

## Discussion

ESCC is a highly invasive and clinically challenging cancer in China, and its molecular basis remains poorly understood. ECRG4 is a novel gene identified and cloned in our laboratory [5,6]. ECRG4 gene is highly conserved among various species, suggesting an important role for ECRG4 in eukaryotic cells [10]. However, its exactly biological function in carcinogenesis is still unclear. Our previous study demonstrated that ECRG4 gene promoter hypermethylation accounted for decreased expression in ESCC, and the low expression of ECRG4 protein in patients with ESCC was associated with poor prognosis [7,8]. These findings were also supported by similar studies of other research groups [11,12]. Furthermore, restoration of ECRG4 expression in ESCC cells inhibited tumor cells growth *in vitro *and *in vivo *[7,8].

In this study, we revealed a novel function of ECRG4 that suppressed tumor cells migration and invasion without affecting cell adhesion ability in ESCC, implicating its potential involvement in tumor development. Li *et al *[13] observed the similar result in glioma consistent with ours. Enhancement in motility and loss of adhesion capacity are advantageous to tumor invasion, which is one main mechanism to cause cancer metastasis. Transformed cells acquire a series of additional malignant traits, such as invasion and metastasis abilities, during tumorigenesis and progression.

It is now generally accepted that transcription factor NF-κB and COX-2 pathway plays a central role between inflammation and carcinogenesis [14,15]. Recently, NF-κB and COX-2 were approved to promote tumor cells migration and invasion [16-23]. Our previous results showed that ECRG4 attenuated NF-κB expression and nuclear translocation and reduced NF-κB target gene COX-2 expression in ESCC [8]. Li *et al *[13] also observed that ECRG4 transfection decreased NF-κB expression in glioma. Therefore, we speculated that NF-κB pathway might be involved in ECRG4-induced decrease of tumor cells migration and invasion in ESCC. However, the detailed molecular mechanism remained to be clarified in subsequent research.

The article "The candidate tumor suppressor gene ECRG4 inhibits cancer cells migration and invasion in esophageal carcinoma" was retracted in 2011. Reasons: duplicated text; duplicate publication.

The cell cycle alteration plays a major role in carcinogenesis. Once the cell cycle regulation balance was broken, it might result in tumorigenesis. Evidence has revealed that many oncogenes and tumor suppressor genes are directly involved in regulation of cell cycle events [24]. In the present research, we discovered for the first time that ECRG4 inhibited cancer cells proliferation and induced cell cycle G1 phase block by up-regulating p21 expression level through p53 mediated pathway in ESCC. It is well known that p21, the critical cyclin-dependent kinase inhibitor, is able to block the cell cycle at G1 phase [25,26]. So the p21 expression upregulation could be the molecular mechanism for the ECRG4-induced cell cycle G1 phase block in ESCC.

Taken together, ECRG4 is a candidate tumor suppressor gene which suppressed cancer cells migration and invasion in ESCC. Furthermore, ECRG4 could also cause cell cycle G1 phase block through the upregulation of p53 and p21 expression levels. Our study indicated that loss of ECRG4 function might play a pivotal role in ESCC carcinogenesis and implied that ECRG4 could be an important therapeutic target for ESCC.

## Abbreviations

ECRG4: esophageal cancer related gene 4; ESCC: esophageal squamous cell carcinoma; NF-κB: NF-kappaB; COX-2: cyclooxygenase 2; GAPDH: glyceraldehyde-3-phosphate dehydrogenase; PBS: phosphate-buffered saline; RT-PCR: reverse transcriptase-polymerase chain reaction.

## Competing interests

The authors declare that they have no competing interests.

## Authors' contributions

LL carried out cell culture, gene transfection, gene functional assays, RT-PCR and Western blotting. CZ and XL analyzed and interpreted data. YZ and SL supervised experimental and wrote the manuscript. All authors read and approved the final manuscript.
